# Histogram Analysis of Diffusion Weighted Imaging in Low-Grade Gliomas: *in vivo* Characterization of Tumor Architecture and Corresponding Neuropathology

**DOI:** 10.3389/fonc.2020.00206

**Published:** 2020-02-25

**Authors:** Georg Alexander Gihr, Diana Horvath-Rizea, Elena Hekeler, Oliver Ganslandt, Hans Henkes, Karl-Titus Hoffmann, Cordula Scherlach, Stefan Schob

**Affiliations:** ^1^Katharinenhospital Stuttgart, Clinic for Neuroradiology, Stuttgart, Germany; ^2^Department for Pathology, Katharinenhospital Stuttgart, Stuttgart, Germany; ^3^Katharinenhospital Stuttgart, Clinic for Neurosurgery, Stuttgart, Germany; ^4^Department for Neuroradiology, University Hospital Leipzig, Leipzig, Germany

**Keywords:** low-grade glioma, apparent diffusion coefficient, histogram analysis, radiomics, histopathology, imaging biomarker

## Abstract

**Background:** Low-grade gliomas (LGG) in adults are usually slow growing and frequently asymptomatic brain tumors, originating from glial cells of the central nervous system (CNS). Although regarded formally as “benign” neoplasms, they harbor the potential of malignant transformation associated with high morbidity and mortality. Their complex and unpredictable tumor biology requires a reliable and conclusive presurgical magnetic resonance imaging (MRI). A promising and emerging MRI approach in this context is histogram based apparent diffusion coefficient (ADC) profiling, which recently proofed to be capable of providing prognostic relevant information in different tumor entities. Therefore, our study investigated whether histogram profiling of ADC distinguishes grade I from grade II glioma, reflects the proliferation index Ki-67, as well as the IDH (isocitrate dehydrogenase) mutation and MGMT (methylguanine-DNA methyl-transferase) promotor methylation status.

**Material and Methods:** Pre-treatment ADC volumes of 26 LGG patients were used for histogram-profiling. WHO-grade, Ki-67 expression, IDH mutation, and MGMT promotor methylation status were evaluated. Comparative and correlative statistics investigating the association between histogram-profiling and neuropathology were performed.

**Results:** Almost the entire ADC profile (p25, p75, p90, mean, median) was significantly lower in grade II vs. grade I gliomas. Entropy, as second order histogram parameter of ADC volumes, was significantly higher in grade II gliomas compared with grade I gliomas. Mean, maximum value (ADCmax) and the percentiles p10, p75, and p90 of ADC histogram were significantly correlated with Ki-67 expression. Furthermore, minimum ADC value (ADCmin) was significantly associated with MGMT promotor methylation status as well as ADC entropy with IDH-1 mutation status.

**Conclusions:** ADC histogram-profiling is a valuable radiomic approach, which helps differentiating tumor grade, estimating growth kinetics and probably prognostic relevant genetic as well as epigenetic alterations in LGG.

## Introduction

Gliomas are primary central nervous system (CNS) tumors originating from sustaining glial cells of the CNS and account for approximately 30 percent of all symptomatic brain neoplasms in adults (1). Based upon histopathologic characteristics like mitotic activity, necrosis, cytological atypia and anaplasia, gliomas are subdivided by the World Health Organization (WHO) into four grades, ranging from WHO grade I—which represents biologically rather benign lesions—to WHO grade IV (2), which entails the most aggressive entities. Only tumors matching the WHO criteria for grade I- and II are classified low-grade gliomas (LGG). Most frequently encountered manifestations of LGG are pilocytic astrocytomas (WHO grade I) and diffuse astrocytomas (WHO grade II). Pilocytic astrocytoma is the most common primary brain tumor in childhood, rarely occurring in adults, which commonly follows an uneventful course. However, malignant transformation has been reported in a number of patients and observation vs. intervention remains an individually challenging decision (3).

Diffuse astrocytoma accounts for the vast majority of LGG in adults and generally exhibits a more protracted course with significantly greater long-term survival compared to high-grade gliomas (HGG) (4). Therefore, and related to the fact that diffuse astrocytomas often occur in eloquent brain regions, a conservative “wait and see”-approach including periodic controls is usually employed as standard management for most of these patients, aiming to avoid disabling surgical morbidity but to preserve functional independence as long as possible. On the contrary, several studies in recent years indicated better prognosis and overall survival of patients after partial or total resection, which has partially led to a paradigm shift in therapy from “watchful waiting” toward early tumor surgery (5–7).

The major obstacle rendering the decision for the optimal personalized therapy very difficult is related to the unpredictable course of the individual LGG.

Therefore, precise recognition of the individual neoplasm including information on its tumor heterogeneity and probable tumor-biological evolution is pivotal.

Magnetic resonance imaging (MRI), offering the highest detail of anatomical as well as functional information in CNS neoplasms has become the gold standard for diagnosis and follow up imaging (8). Among the variety of functional imaging techniques like spin labeling, spectroscopy, perfusion weighted imaging etc., especially diffusion-weighted imaging (DWI) has gained significant importance for assessment of brain tumors (9).

By mapping the diffusibility of water molecules in biological tissues through apparent diffusion coefficient (ADC) maps (10), DWI allows assessment of the underlying microscopic architecture of the examined tissue (11). In context of glioma imaging, DWI including ADC-mapping were shown to be especially valuable for tumor grading and the differentiation of LGG from HGG (12), for assessment of prognosis (13), for estimation of tumor growth potential (14) and the differentiation of gliomas from other, morphologically indistinguishable lesions (15).

However, most of the DWI studies investigated simple, mostly two-dimensional region-of-interest-based estimations of the ADC, neither accounting for the three-dimensional complexity of the tissue nor considering all parameters of the ADC histogram. As introduced by Just and coworkers (16), histogram analysis can provide more than first order histogram characteristics, which basically represent specific proportions of one investigated value (in our case the ADC). Those second order characteristics—kurtosis, skewness, and entropy—describe more complex aspects of the (ADC-) distribution and its particular shape, which notoriously facilitate the assessment of the microarchitecture of the particular lesion. The entropy of a histogram profile for example, describing the degree of randomness of the respective distribution, has been established as an important biomarker reflecting tumor heterogeneity in numerous studies (17–19). Interestingly, even the entropy of simple T1-post-contrast image histograms is able to reflect tumor characteristics like mitotic activity to a limited extent (20).

Therefore, our study aimed to evaluate whether whole tumor histogram analysis of ADC maps can (I) differentiate WHO grade I and WHO grade II tumors, (II) predict the proliferative potential of those neoplasms and (III) predict the presence of prognostic relevant MGMT (methylguanine-DNA methyl-transferase) promotor methylation and IDH (isocitrate dehydrogenase) mutation status.

## Patients, Procedures, and Methods

### Ethics Approval

The study was approved by the ethics committee of the medical council of Baden-Württemberg (Ethik-Kommission Landesärztekammer Baden-Württemberg, F-2017-047).

### Patients Collective

The institutional radiological information system (RIS) was searched for patients with the diagnosis glioma and primary brain tumor. Histopathologic diagnosis, Ki-67 proliferation index, IDH-1 mutation status and MGMT promotor methylation status were obtained by searching the hospital patient database. Forty-two patients were identified between 01/2012 and 02/2017, all of which had at least diagnostic biopsy or even surgical removal of the tumor in our hospital and subsequent neuropathological workup. Only patients who received pretreatment MRI scans with sufficient DWI were included. MRI examinations of patients indicating hemorrhage, significant calcifications or artificial MRI data due to other causes were excluded, since these conditions severely influence quantification, and hence, produce incorrect ADC values. Therefore, only 26 patients (12 females, 14 males; ranging from 5 to 58 years with a mean age of 34.2 years) were included in our retrospective analysis: 7 patients with the diagnosis of pilocytic astrocytoma (WHO grade I), 19 patients with the diagnosis of diffuse astrocytoma (WHO grade II); 15 out of 26 patients with IDH-1 mutation and 8 out of 26 patients with IDH-1 wildtype (of 3 patients no IDH-1 mutation status was available); 9 out of 26 patients patients with MGMT promotor methylation and 6 out of 26 patients with unmethylated MGMT promotor (of 11 patients no MGMT promotor methylation status was available); of 2 out of 26 patients no Ki-67 proliferation index was available.

### MRI Specifics

For all patients MRI of the brain was performed using a 1.5 T device (MAGNETOM Aera and MAGNETOM Symphony Tx/Rx CP head coil, Siemens, Erlangen, Germany). The imaging protocol included the following sequences:

1. Axial T2 weighted (T2w) turbo spin echo (TSE) sequence (TR/TE: 5390/99, flip angle: 150°, slice thickness: 5 mm, acquisition matrix: 512 x 291, field of view: 230 x 187 mm);
2. Axial DWI (readout-segmented, multi-shot EPI sequence; TR/TE: 5500/103, flip angle 90°, slice thickness: 5 mm, acquisition matrix: 152 x 144, field of view: 230 x 230 mm) with b values of 0 and 1,000 s/mm^2^. ADC maps were generated automatically by the implemented software package.

All images were available in digital form and analyzed by two experienced radiologists (DHR, SS) without knowledge of the histopathological diagnosis on a PACS workstation (Impax EE R20 XII).

### Histogram Profiling of ADC Maps

ADC maps and T2 weighted images were exported from our institutional archive in DICOM format *via* the aforementioned AGFA PACS. Whole lesion histogram profiling was performed by using a custom-made DICOM image analysis tool (programmed by N.G. using Matlab, The Mathworks, Natick, MA): T2 weighted images were loaded into a graphical user interface (GUI) to tag the tumor suspected lesion of each patient in all respective MRI sections. All regions of interest (ROIs) were then automatically co-registered with the corresponding ADC maps and the whole lesion histogram profile was consecutively calculated, providing the following set of parameters: ADCmean, ADCmin, ADCmax, ADCp10, ADCp25, ADCp75, ADCp90, ADCmodus, ADCmedian, ADC standard deviation (SD), Skewness, Kurtosis, and Entropy.

### Neuropathology

All tumor specimens were used for neuro-histological confirmation of the diagnosis. The tumor samples, obtained either by stereotactic biopsy, partial or complete resection were formalin-fixed and paraffin-embedded for histopathologic diagnostics, immunohistochemistry and PCR sequencing. The embedded samples were sectioned at 3 μm and stained by hematoxylin and eosin (H&E). Immunhistochemistry was performed with specific antibodies against IDH1-R132H (dilution 1:20, product no. DIA-H09; Dianova, Hamburg, Germany) and Ki67 M7240 (dilution 1: 800; Dako Denmark A/S, Glostrup, Denmark). The histopathological images were digitalized with a Leica microscope, carrying a DFC290 HD digital camera and LAS V4.4 software (Leica Microsystems, Wetzlar, Germany). Sample sections for immunohistochemistry and PCR sequencing were analyzed histologically for presence of viable tumor infiltration and absence of necrotic areas and hemorrhage. In case of IDH1 immunohistochemistry a strong cytoplasmic staining was interpreted as positive result. Tumor proliferation index was estimated by dividing the number of specifically stained (Ki-67 positive) cell nuclei by all nuclei. The area showing the highest number of positive cell nuclei was selected in each case.

To determine the methylation status of the MGMT gene, tumor DNA was isolated from micro-dissected 10 μm sections from the paraffin-embedded tissue blocks using the Maxwell® RSC FFPE Plus DNA Kit AS1720 (Promega, USA) with a Maxwell® RSC Instrument (Promega, USA), followed by conversion of unmethylated cytosine residues to uracil by bisulfite treatment using the EpiTect® Bisulfite Kit (QIAGEN, Germany), each step according to the manufacturer's procedures. Bisulfite-converted DNA was amplified in a PCR reaction and the methylation status was determined by pyrosequencing according to the manufacturer's protocol using the Therascreen MGMT Pyro® Kit (QIAGEN, Germany), testing 4 CpG islands (chromosome 10, Exon 1, range 131265519-131265537, CGACGCCCGCAGGTCCTCG). Methylation percentage of 10% and higher was considered as methylation positive.

### Statistical Analysis

Statistical analysis including graphics creation was performed using GraphPad Prism 8 (GraphPad Software, San Diego, CA, USA). In a first step, DWI data and histopathological information were investigated using descriptive statistics. In a second step, data was tested for Gaussian distribution using the Shapiro-Wilk-Test. *T*-test was performed to compare evaluated, normally distributed parameters of DWI histogram profiling between grade I and grade II astrocytoma. Also, normally distributed DWI histogram profiling parameters between IDH mutated and IDH wildtype gliomas as well as between MGMT promotor methylated and unmethylated gliomas were compared using unpaired *T*-test. Mann-Whitney-U Test was performed to compare parameters exhibiting a non-Gaussian distribution between grade I and grade II, between IDH mutation positive and negative as well as between MGMT promotor methylated and unmethylated astrocytomas. Finally, correlation analysis for normally distributed parameters was performed using Pearson Correlation Coefficient. In case of non-Gaussian distribution, Spearman-Rho Rank-Order Correlation was calculated. *p*-values < 0.05 were taken to indicate statistical significance in all instances. Finally, to assess the accuracy of ADC volume histogram profiling, receiver operating characteristics (ROC) curve analysis was performed and the respective area under the curve (AUC) was calculated as well as Youden's Index for those ADC parameters with the best test accuracy to estimate possible cut-off values.

## Results

Figure 1 demonstrates examples of cranial MRI from patients with WHO grade I (upper row) and WHO grade II astrocytoma (lower row) including the corresponding whole tumor ADC histogram, H&E staining and Ki-67 immunohistochemistry.

**Figure 1:** Compares representative MRI sections, the corresponding whole tumor ADC histogram, H&E staining, and Ki-67 immunohistochemistry of a grade I **(A–D)** and a grade II glioma **(E–H)**. The first image of the upper case shows a T2 weighted turbo-spin-echo (TSE) sequence of a grade I glioma, originating from the right thalamus with intraventricular tumor mass in the third ventricle and consecutive hydrocephalus **(A)**. The first image of the lower case displays a T2 weighted TSE sequence of a grade II diffuse astrocytoma located in the right frontal and parietal lobe with distinct mass effect **(E)**. The second images of each row show the ADC histograms (**B,F**; x-axis: ADC values in incremental order, y-axis: number of voxels) followed by H&E staining and Ki-67 immunohistochemistry on the right side **(C–D**, **G–H)**. For the first case (pilocytic astrocytoma), a proliferation index of 1% was calculated. In the second case (diffuse astrocytoma), proliferation index was 5%.

The results of the descriptive analysis of DWI data of all investigated gliomas are summarized in Table 1. Shapiro-Wilk-Test revealed Gaussian distribution for ADCmean, ADCmin, ADCmax, ADCp10, ADCp25, ADCp75, ADCp90, ADCmodus, ADCmedian, ADC SD, Entropy and Ki-67 (all *p* < 0.05). Non-Gaussian distribution was determined for Kurtosis and Skewness.

**Table 1:** DWI histogram profiling parameters of all investigated low-grade gliomas.

**Parameters**	**Mean ± standard deviation**	**Minimum**	**Maximum**
ADC_mean_, × 10^−5^ mm^2^s^−1^	148.73 ± 31.41	88.10	230.91
ADC_min_, × 10^−5^ mm^2^s^−1^	53.75 ± 24.97	0.10	93.20
ADC_max_, × 10^−5^ mm^2^s^−1^	260.53 ± 57.92	159.30	352.80
P10 ADC, × 10^−5^ mm^2^s^−1^	109.99 ± 15.15	71.60	136.80
P25 ADC, × 10^−5^ mm^2^s^−1^	129.33 ± 26.08	77.40	203.60
P75 ADC, × 10^−5^ mm^2^s^−1^	167.85 ± 41.31	98.10	272.70
P90 ADC, × 10^−5^ mm^2^s^−1^	185.28 ± 46.16	107.20	279.10
Median ADC, × 10^−5^ mm^2^s^−1^	148.91 ± 35.51	86.50	263.30
Mode ADC,	153.24 ± 45.35	84.00	276.90
SD ADC, × 10^−5^ mm^2^s^−1^	30.11 ± 13.57	12.76	64.11
Kurtosis	4.23 ± 2.71	2.00	11.20
Skewness	0.32 ± 0.87	−1.35	2.47
Entropy	5.19 ± 0.69	3.79	6.19

Statistical significant differences between grade I and grade II astrocytomas were identified for the following set of ADC histogram parameters: ADCmean, ADCmax, ADCp25, ADCp75, ADCp90, ADCmedian, ADC SD, and Entropy (all *p* < 0.05). Mean values of ADC fractions, except the lowest percentile (ADCp10), the minimum values (ADCmin) and the ADC modus, were all significantly lower in the WHO grade II group, whereas Entropy was significantly greater in WHO grade II gliomas compared to grade I gliomas. The standard deviation (SD) of ADC histogram profiles of grade II astrocytomas was significantly lower than in the group of grade I tumors. Differences in Ki-67 expression, representing the actively proliferating tumor fraction, also achieved statistical significance, with increased values in the WHO grade II group. Furthermore, significant differences between MGMT promotor methylated and unmethylated gliomas were identified for ADCmin, being increased in unmethylated gliomas. Comparison of ADC histogram profiles of IDH-1 mutated and IDH-1 wildtype astrocytomas revealed significant differences for Entropy, with higher values in case of muted IDH-1. For reasons of comprehensibility and clarity, results of the comparative statistical analysis are summarized in Tables 2–4. Figures 2A–H shows significant differences in ADC histogram profile parameters between WHO grade I and II astrocytomas, Figures 2I,J illustrates differences of ADC Entropy and ADCmin considering IDH-1 mutation status and MGMT promotor methylation status of the investigated gliomas.

**Table 2:** Comparison of DWI histogram profiles and Ki-67 index between grade I and grade II glioma.

**Parameters**	**WHO grade 1**		**WHO grade 2**		***T*-test**
	**Mean** **±** **SD**		**Mean** **±** **SD**		***p*-values**
ADC_mean_, × 10^−5^ mm^2^s^−1^	171.90	36.80	140.20	26.25	**0.0221**
ADC_min_, × 10^−5^ mm^2^s^−1^	61.67	32.25	50.84	22.82	0.3463
ADC_max_, × 10^−5^ mm^2^s^−1^	315.30	34.31	240.40	53.46	**0.0022**
P10 ADC, × 10^−5^ mm^2^s^−1^	116.90	9.53	107.40	16.60	0.1692
P25 ADC, × 10^−5^ mm^2^s^−1^	146.4	31.88	123.10	22.12	**0.0452**
P75 ADC, × 10^−5^ mm^2^s^−1^	197.70	51.56	156.90	33.25	**0.0251**
P90 ADC, × 10^−5^ mm^2^s^−1^	222.50	52.55	171.60	37.69	**0.0112**
Median ADC, × 10^−5^ mm^2^s^−1^	172.00	47.97	140.40	27.76	**0.0460**
Mode ADC, × 10^−5^ mm^2^s^−1^	179.70	67.76	143.50	32.65	0.0753
SD ADC, 10^−5^ mm^2^s^−1^	42.16	14.76	25.67	10.78	**0.0045**
Kurtosis	5.50	3.91	3.76	2.16	0.2542
Skewness	0.70	1.25	0.18	0.70	0.2307
Entropy	4.72	0.67	5.37	0.65	**0.0350**
Ki-67	3.00	1.73	5.41	2.58	**0.0340**

*Values displayed in bold indicate findings of statistical significance (p ≤ 0.05)*.

**Table 3:** Comparison of DWI histogram profiles between low-grade gliomas with and without MGMT promotor methylation.

**Parameters**	**MGMT promotor methylation positive**		**MGMT promotor methylation negative**		***p*-values**
	**Mean** **±** **SD**		**Mean** **±** **SD**		
ADC_mean_, × 10^−5^ mm^2^s^−1^	142.30	27.35	141.1	25.71	0.9286
ADC_min_, × 10^−5^ mm^2^s^−1^	41.76	19.13	62.62	24.47	**0.033**
ADC_max_, × 10^−5^ mm^2^s^−1^	246.40	55.41	226.70	68.03	0.5480
P10 ADC, × 10^−5^ mm^2^s^−1^	108.60	17.04	106.90	15.41	0.8429
P25 ADC, × 10^−5^ mm^2^s^−1^	125.40	23.76	121.20	18.74	0.7201
P75 ADC, × 10^−5^ mm^2^s^−1^	159.80	32.75	157.20	36.64	0.8861
P90 ADC, × 10^−5^ mm^2^s^−1^	173.10	34.43	177.90	46.59	0.8202
Median ADC, × 10^−5^ mm^2^s^−1^	143.50	29.87	139.10	24.84	0.7678
Mode ADC, × 10^−5^ mm^2^s^−1^	145.10	35.54	139.10	22.84	0.7224
SD ADC, × 10^−5^ mm^2^s^−1^	25.34	7.88	28.93	16.00	0.5697
Kurtosis	3.25	0.81	3.50	2.21	0.6889
Skewness	0.02	0.38	0.40	0.95	0.6070
Entropy	5.62	0.49	4.97	0.80	0.0719

*Values displayed in bold indicate findings of statistical significance (p ≤ 0.05)*.

**Table 4:** Comparison of DWI histogram profiles between low-grade gliomas with and without IDH-1 mutation.

**Parameters**	**IDH-1 mutation**		**IDH-1 wildtype**		
	**Mean** **±** **SD**		**Mean** **±** **SD**		***p*-values**
ADC_mean_, × 10^−5^ mm^2^s^−1^	143.10	22.50	148.30	34.58	0.6678
ADC_min_, × 10^−5^ mm^2^s^−1^	53.17	25.88	65.08	14.91	0.2465
ADC_max_, × 10^−5^ mm^2^s^−1^	241.70	53.59	278.20	60.52	0.1514
P10 ADC, × 10^−5^ mm^2^s^−1^	110.40	15.21	108.90	18.47	0.8390
P25 ADC, × 10^−5^ mm^2^s^−1^	126.00	19.93	124.80	24.53	0.8987
P75 ADC, × 10^−5^ mm^2^s^−1^	158.80	27.96	171.90	49.04	0.4201
P90 ADC, × 10^−5^ mm^2^s^−1^	174.70	30.90	191.60	56.67	0.3601
Median ADC, × 10^−5^ mm^2^s^−1^	143.20	24.73	144.30	32.66	0.9325
Mode ADC, × 10^−5^ mm^2^s^−1^	145.50	30.31	153.50	57.96	0.6623
SD ADC, × 10^−5^ mm^2^s^−1^	25.91	9.84	33.38	13.75	0.1457
Kurtosis	3.51	1.42	4.97	3.87	0.9748
Skewness	0.15	0.75	0.77	0.92	0.1688
Entropy	5.5	0.63	4.75	0.69	**0.0144**

*Values displayed in bold indicate findings of statistical significance (p ≤ 0.05)*.

**Figure 2:** Provides boxplots of statistically significant differences between the diffusion profile of grade I and grade II gliomas **(A–H)** as well as between IDH-1 mutation status **(I)** and MGMT promotor methylation status **(J)** positive and negative tumors. The last image **(K)** shows the significant correlation between ADCmax of the whole tumor ADC histograms and the proliferation index Ki-67, the set of parameters with the strongest correlation (r = −0.5218, *p* = 0.0089).

Correlative statistics revealed significant correlations (*p* < 0.05) between Ki-67 and ADCmean, ADCmax, ADCp10, ADCp75, ADCp90 as well as ADC SD. Table 5 summarizes the complete results of the correlative analysis. The scatter plot graphically demonstrating the association of ADCmax and Ki-67, the set of parameters with the strongest correlation (*r* = −0.5218, *p* = 0.0089), is shown in Figure 2K.

**Table 5:** Correlations between DWI histogram profile parameters and Ki-67 in all investigated gliomas.

**DWI histogram profile parameters**	**Ki-67**
ADC_mean_, × 10^−5^ mm^2^s^−1^	***r*** **=** **−0.4389**
	***p*** **=** **0.0319**
ADC_min_, × 10^−5^ mm^2^s^−1^	*r* = **–**0.03701
	*p* = 0.8637
ADC_max_, × 10^−5^ mm^2^s^−1^	***r*** **=** **−0.5218**
	***p*** **=** **0.0089**
ADCp10, × 10^−5^ mm^2^s^−1^	***r*** **=** **−0.4187**
	***p*** **=** **0.0417**
ADCp25, × 10^−5^ mm^2^s^−1^	*r* = **–**0.3767
	*p* = 0.0696
ADCp75, × 10^−5^ mm^2^s^−1^	***r*** **=** **−0.4328**
	***p*** **=** **0.0347**
ADCp90, × 10^−5^ mm^2^s^−1^	***r*** **=** **−0.4512**
	***p*** **=** **0.0269**
ADCMedian, × 10^−5^ mm^2^s^−1^	*r* = **–**0.3759
	*p* = 0.0702
ADCModus, × 10^−5^ mm^2^s^−1^	*r* = **–**0.3179
	*p* = 0.1011
SD ADC, × 10^−5^ mm^2^s^−1^	***r*** **=** **−0.4475**
	***p*** **=** **0.0283**
Kurtosis	*r* = 0.1312
	*p* = 0.5412
Skewness	*r* = 0.0885
	*p* = 0.6810
Entropy	*r* = 0.2186
	*p* = 0.3048

*Values displayed in bold indicate findings of statistical significance (p ≤ 0.05)*.

Furthermore, AUC values were calculated for each of the evaluated parameters exhibiting statistically significant differences between grade I and grade II astrocytomas with the following results (CI: confidence interval): ADCmean [AUC = 0.737, (CI: 0.502–0.972), *p* = 0.067], ADCmax [AUC = 0.895, (CI: 0.768–1.000), *p* = 0.0024], ADCp25 [AUC= 0.722, (CI: 0.494–0.949), *p* = 0.088], ADCp75 [AUC = 0.744, (CI: 0.518–0.970), *p* = 0.060], ADCp90 [AUC = 0.797, (CI: 0.576–1.000), *p* = 0.022], ADCmedian [AUC = 0.729, (CI: 0.494–0.965), *p* = 0.078], ADC SD [AUC = 0.805, (CI: 0.613–0.996), *p* = 0.019] and Entropy [AUC = 0.752, (CI: 0.559–0.945), *p* = 0.053]. Figure 3 displays the corresponding ROC of ADCmax, the parameter with the best accuracy. Finally, Youden's Index for ADCmax was calculated to estimate the most promising cut-off value revealing the following result: ADCmax values of 0.002632 and greater indicate grade I astrocytoma (sensitivity: 0.684, specificity: 1.00).

**Figure 3:** Provides the receiver operating characteristics (ROC) curve of ADCmax, the parameter with the best accuracy in terms of differentiating grade I and grade II gliomas.

## Discussion

Despite the revision of the WHO classification of CNS tumors in 2016, which integrated a panel of molecular parameters (2), general histology obtained by light microscopy still remains a major pillar in the glioma grading system. As a consequence, presurgical determination of a tumor's microarchitecture including the identification of potential hot spots, resembling areas of above-average increased proliferation, as targets for biopsy or partial resection is pivotal.

In this regard, our study showed significantly lower values in a variety of the ADC histogram items, more specifically ADCmean, ADCmax, ADCp25, ADCp75, and ADCp90 as well as ADCmedian when comparing grade II with grade I LGG. This finding is in line with earlier reports on the connection between ADC and decreased extracellular space related to increased proliferation and subsequently cellularity (21–24), inherently restricting Brownian motion of extracellular water molecules. As a substantial corroboration, our study confirmed significant differences in Ki-67 expression-based proliferation index when comparing WHO grade I and WHO grade II LGG, varifying higher values in grade II gliomas.

Considering those results, diffusion profiles are valuable tools in addition to anatomic imaging to identify subtle, but biologically distinct tumor compartments in LGG.

Increasing body of evidence suggests the superior value of additionally using the second order histogram dimensions skewness, kurtosis and entropy of the ADC-continuum, for better reflection of tumor heterogeneity and associated tumor-biology (16, 17, 20, 21, 25–32). In this regard, our results show the significant differences of ADC-entropy in grade I vs. grade II LGG, with higher values being associated with higher tumor grade. A comparable relation has been shown in other tumor entities (29). It is indisputable, that higher tumor grades entail increased heterogeneity at the microstructural level, which is accurately reflected by ADC histogram profiles derived from LGG in our analysis.

Low-grade gliomas (LGG) often harbor mutations in one of both genes for IDH. A growing body of evidence indicates that these mutations are at least co-causative for glioma-genesis (33) and therefore represent promising future therapeutic targets. So far, IDH mutation status is a well-established and important prognostic factor in low-grade glioma with better prognosis and survival in case of mutated IDH genes compared to wild-type genes (34–36). The presented ADC histogram analysis elucidates the (so far unreported) potential of ADC entropy to distinguish IDH-mutated and IDH-wild-type LGG. The meaningfulness of this feature cannot be proven by this singular report, but it indicates the potential value of this imaging biomarker and should stimulate further investigations.

A second, equally important molecular property in gliomas bearing great prognostic relevance is the MGMT promotor methylation status. MGMT is a very important DNA repair enzyme. Its expression may be silenced by methylation of its promotor during tumor development, which in turn increases the anti-proliferative effect of alkylating chemotherapeutics. MGMT promotor methylation is associated with an improvement in overall survival (37) in patients suffering from glioblastoma and influences the overall survival of patients with LGG (38). A number of studies investigated the potential of ADC histogram parameters obtained by presurgical MRI for prediction of the MGMT promotor methylation status in glioblastoma, but the results concurrently remain ambiguous (39–43). Also, studies investigating ADC histogram profiling regarding MGMT promotor methylation status in low-grade glioma are completely lacking. Our study shows a significant difference in ADCmin values of LGG with vs. LGG without MGMT promotor methylation. This association is definitely interesting and has the potential to substantiate the importance of histogram profiling for presurgical assessment of individual brain neoplasms, but certainly requires confirmation in a larger cohort.

Finally, significant inverse correlations between Ki-67 expression and ADCmean, ADCmax and the percentiles ADCp10, ADCp75, and ADCp90 were demonstrated. These results are in line with previously published reports on primary CNS lymphomas and meningiomas, proving an inverse correlation between different ADC fractions and Ki-67 expression (25, 29). As discussed above, high Ki-67 expression is a hallmark of increased proliferative activity in neoplastic tissue, naturally resulting in increased cellular density and restricted interstitial diffusion, which is reflected by altered ADC values. In contrast to the first order histogram characteristics, none of the second order characteristics, namely entropy, kurtosis and skewness, showed a significant correlation with Ki-67 expression.

Our study suffers from the following relevant limitations. First of all, it is only a retrospective investigation of a relatively small patient cohort. Furthermore, only data from 1.5-T MRI systems were available, which inevitably leads to lower signal to noise ratios of the MRI data, necessitating acquisition of MRI pictures with smaller pixel matrix and therefore reduced spatial information compared to examinations with a higher field strength. Finally, ADC was calculated by using only 2 b values (0 and 1,000 s/mm^2^) and small vessel perfusion could therefore have an impact on ADC values in our patient collective.

## Conclusion

ADC histogram profiling of LGG provides first and second order characteristics allows to draw inferences about the proliferative activity of the lesion at hand and facilitates differentiation of grade I from grade II neoplasms, which may be important for risk stratification especially in cases of extended tumor infiltration or tumors in eloquent brain areas associated with high perioperative morbidity. Furthermore, our results indicate that ADC histogram profiling enables to draw conclusions about the prognostic relevant IDH mutation status and MGMT promotor methylation status in LGG. As a consequence, inclusion of ADC histogram profiling for presurgical definition of morphologically inapparent, tumor-evolutional significant compartmentation is recommended to increase the accuracy of diagnosis and prognosis and to help the treating physician to identify the most appropriate treatment strategy.

## Data Availability Statement

Data of the descriptive analysis, group comparisons, and correlative analysis are provided in the supplement. Additional data on the individual case level can be requested from the corresponding author.

## Ethics Statement

The studies involving human participants were reviewed and approved by ethics committee of the medical council of Baden-Württemberg (Ethik-Kommission Landesärztekammer Baden-Württemberg, F-2017-047). The patients/participants provided their written informed consent to participate in this study.

## Author Contributions

GG and SS conceived and planned the present study and supervised the project. GG and DH-R were responsible for data acquisition. GG performed statistical analyses and took lead in writing the manuscript. EH was responsible for histopathological workup and figures. HH, K-TH, OG, and CS contributed to the interpretation of the results, provided critical feedback and helped shape the research and manuscript.

### Conflict of Interest

The authors declare that the research was conducted in the absence of any commercial or financial relationships that could be construed as a potential conflict of interest.
